# A New Data Model for the Privacy Protection of Medical Images

**DOI:** 10.1155/2022/5867215

**Published:** 2022-07-09

**Authors:** Lijing Ren, Denghui Zhang

**Affiliations:** ^1^Cyberspace Institute of Advanced Technology, Guangzhou University, Guangzhou 510006, China; ^2^School of Traffic and Transportation, Shijiazhuang Tiedao University, Shijiazhuang 050043, China

## Abstract

Benefiting from the intelligent Medical Internet of Things (IoMT), the medical industry has dramatically improved its quality and productivity. The transmission of biomedical data in an open and untrusted network poses a new challenge to the privacy protection of patient information. The low processing power of IoMT limited the application of traditional encryption to protect sensitive data. In this paper, we developed a new data protection model for medical images. The model uses visual cryptography (VC) to store biomedical data in a separate database, which can transfer the sensitive data of patients simply and securely. To alleviate the degradation of biomedical recognition performance caused by VC-based noise, we further use transfer learning to train an optimized neural network. The experimental results show that this proposed method provides privacy in the IoMT environment and maintains the high accuracy of biomedical recognition.

## 1. Introduction

The Internet of Things (IoT) is a paradigm change which jointly optimized previously competing sensing and communication operations via the same hardware and spectrum resource [1]. It is widely used in healthcare, including medical devices, sensors, and healthcare systems [2]. Along with the interconnection of medical devices and healthcare services, it is now becoming increasingly important to understand the emerging IoT-based healthcare systems [3]. As a promising cellular network, IoMT is an important future research direction towards further combining with artificial intelligence (AI) technologies to realize from Internet of everything to the intelligent interaction of patients and medical sensors [4].

Biomedical data are widely used perceptual information transmitted on the Internet [5]. Security issues with the technology that stores, sends, and receives medical data can lead to the exposure of personal healthcare information (PHI) online. Recently, researchers from a vulnerability analysis company found that there were 600 unsafe PACS (Picture Archiving and Communications Systems) servers on the public network, which caused 400 million medical radiological images to be leaked, involving about 24.3 million patient records [6].

Personal medical images should be kept confidential to protect the patient's privacy from being compromised. Theoretically, modern public-key cryptography and watermarking can be used to encrypt medical images [7]. However, due to the limitation of image data itself, the traditional encryption scheme based on text cannot be directly applied to electronic image data [8]. Besides, considering the constraints of real-time data acquisition, a satisfactory level of security is to be achieved with a fast and lightweight encryption method. Medical image encryption can be divided into storage encryption and transmission encryption [2]. In the process of storage, image hiding and image encryption can be used for the information security of images. In the process of image transmission, image communication encryption technology can be adopted, and the privacy of patients can be ensured by the encryption technology in communication. However, these methods often require a lot of time to perform complex cryptographic operations, and the communicating parties need to spend extra steps to establish an encrypted channel [9]. These characteristics have hindered the spread of medical image encryption.

Visual Cryptography (VC) [10] is a secret-sharing technology for images. It removes the complex mathematical operation and key dependence in traditional public-key cryptography and digital watermarking. VC only needs a simple Boolean operation to encrypt and decrypt images. If the encrypted sharing is printed out, the image can be restored by simple superposition, even without any digital devices. VC provides an efficient encryption scheme for computing-limited scenarios such as medical image transmission. However, there still exist problems in VC including pixel expansion and noise shares which are suspicious and vulnerable.

In this paper, we propose a new VC-based data model to protect the privacy of medical images in transmission [11]. Firstly, we propose a meaningful and friendly VC scheme without pixel expansion aiming at the limitations of the traditional VCSs (VC Schemes). After that, we divide a sensitive image into several unrelated images using the proposed VC scheme and transmit and store them independently, so as to archive the safe transmission of medical images. Then, to issue the problem that the noise of the decrypted image interferes with the recognition performance, we obtain the pretraining weights from large-scale datasets and transfer them to VC-based lossy dataset recognition networks by the transfer learning method [12]. The contributions of this paper are as follows:

1. We propose a novel user-friendly visual cryptography mechanism without pixel expansion.
2. We propose a safe and efficient transmission method of medical images using the secret-sharing characteristics of visual cryptography.
3. We propose a high-precision neural network recognition method for encrypted data sets.

## 2. Related Work

### 2.1. Biomedical Recognition

In the past decades, biomedical recognition technology has made remarkable progress [13]. The core of the traditional feature recognition methods lies in the well-designed representation. The recognition performance of traditional machine learning algorithms such as SVM (Support Vector Machines) and PCA (Principal Component Analysis) gradually reached a bottleneck. So, researchers shift their focus to recognition algorithms based on deep learning [14, 15]. The classic CNN (Convolution Neural Networks) integrates methods including convolution network and pooling method to improve the accuracy of image recognition [16, 17].

There have been a lot of landmark achievements in the field of biomedical recognition. This section only discusses the research progress of metric learning involved [18]. Feature recognition is a process of similarity measurement. To solve the problem that the loss function of softmax leads to the lack of boundaries of training targets, Yann et al. [14] introduced contrastive loss as the loss function to train a network in the process of data dimensionality reduction, to increase the Euclidean distance of different types of samples and speed up the convergence speed of training. Based on the same principle, Schroff et al. [19] introduced the triplets loss function to embedding images into multidimensional Euclidean space to further improve the recognition accuracy. Space ensures that the embedding distance of a certain image is close to its similar image, and the distance from other different types of images is far enough. Snell et al. [20] turned the classification problem of image recognition into the nearest neighbor problem of embedding. In this model, each class has a prototype expression, and the prototype of this class is the average value of a training set in the embedding space. In prediction, the class label of images can be archived by calculating the softmax of the distance between the test sample and each class prototype.

### 2.2. Visual Cryptography (VC)

Visual cryptography is an image-oriented (*k*, *n*) threshold secret-sharing scheme first proposed by Base et al. [21]. In this scheme, a secret black and white image is divided into *n* shares, and then the shares are distributed to *n* participants. The threshold characteristic of VC makes it impossible to restore the secret image unless shares held by  *k* (*k* < *n*) or more participants are superimposed together.

Although VCS eliminates the complicated operation process of traditional encryption technologies, there are still two major defects. The first is pixel expansion. Pixel expansion means that the size of the secret image cannot be too large; otherwise, it will be difficult to align and superimpose the printed shares. The second disadvantage of VC is that the contrast of the restored image decreases, while the human eye can only recognize the secret image with sufficient contrast. Many improvement schemes have been proposed at present. But these methods are all at the expense of other characteristics of visual cryptography [22, 23]. For example, VCSs based on probability or block technology solve the problem of pixel expansion; it has the problem of quality loss [8]. The vertical expansion method, although it can improve the contrast, often needs to share multiple images (maybe as many as 100), and smart devices are often sensitive to network traffic [24]. Although high-quality VCS can be realized by using XOR operation and QR code, it often needs additional noise shares [23]. The size of standard QR codes and the capacity of error correction codes are limited, which cannot meet the needs of image transmission [25].

## 3. Methods

The section organically combines VC with biomedical features and adopts distributed storage and transfer learning methods to realize privacy protection and high-precision identification of biomedical features.

### 3.1. Expansion-Free EVCS

To solve the problem that noised shares are vulnerable to attack, this subsection will use meaningful sharing instead of noised shares, which further increases the difficulty of VCS construction. Block encryption and halftone technology can only partially solve the problem of contrast loss. How to propose a novel VCS with no expansion and high contrast will be the key to this topic.

The traditional VC adopts a pixel-by-pixel encryption method. For a single white (*w*) or black pixel (*b*), there is a corresponding encryption matrix set *C*_0_ (*C*_1_), where the matrix consists of *n* × *m* Boolean values. As shown in Figure 1, in the (2, 2)-VCS with 4-pixel extension ((*m*=4)), *C*_0_ and *C*_1_ can be obtained by random permutation of the columns of the two basis matrices *S*_0_ and *S*_1_. For white (or black) pixels in the image, a matrix is randomly selected from *C*_0_ or *C*_1_ in the encryption process, and each row of pixels in the matrix is allocated to the corresponding Share_*i*_,  *i* ≤ 2. Each pixel of the secret image is coded as *n*=2 rows in the matrix and distributed to 2 participants, each row containing 4 subpixels.

The extended VCS (EVCS) [26] adopts meaningful images as covers rather than noise-like images to encrypt images. Compared with VCS, this mechanism can avoid suspicions caused by noise images, and shares are more convenient for management. Meaningful shares can be publicly transmitted without revealing the information of secret images.  Figure 2 illustrates the encryption and decryption of a simple (2, 2)-EVCS. The scheme represents a black pixel with subpixels consisting of 4 black pixels in the secret image and subpixels consisting of 3 black pixels and 1 white pixel in cover images, while it represents a black pixel with subpixels consisting of 3 black pixels and 1 white pixel in the secret image, and subpixels consisting of 2 black pixels and 2 white pixels in cover images. Because the contrast of white subpixel and black in the secret image is different, human eyes can still reveal the information in the secret image. The contrast in the cover images is also different, so the human eye can also see the secret information; that is, the cover images are meaningful. In the traditional VCS, the contrast of black and white subpixels is the same; thus we cannot distinguish them.

Let *s*_*c*1*c*2_^*s*^ denotes a basis matrix where the secret pixel is *s*; pixels in two shares are *c*1 and *c*2. We use 1 to denote a black pixel and 0 to denote a black pixel. So, the recovery Boolean operation alters to AND from OR. Note that the indication may be opposite to the common, which uses 1 to denote black pixels and 0 to denote white pixels since white is often the background color. If we want to encrypt a black secret pixel (0), we can use subpixels in any row on the left of Figure 2 to encode shares. Taking the first row, for example, this row consists of 3 black pixels and 1 white pixel, that is,

(1) $$\begin{array}{c} S_{b}^{\text{bb}}=\left[\begin{array}{cccc} 0 & 1 & 0 & 0\\ 1 & 0 & 0 & 0 \end{array}\right],\\ S_{w}^{\text{bb}}=\left[\begin{array}{cccc} 0 & 1 & 0 & 0\\ 0 & 1 & 0 & 0 \end{array}\right]. \end{array}$$

We can permute the columns of the basic matrix to generate candidates encoding for the secret black pixel. If an attacker gets a black subpixel *c*1=[0 1 0 0] from a cover, it still is impossible to infer the corresponding secret pixel in the secret image. When the subpixel at the corresponding position in another cover is *c*2=[1 0 0 0], the superimposed subpixel will be *r*=[0 0 0 0], and the superimposed pixel is black. When *c*2=[0 1 0 0], the superimposed pixel *r*=[0 1 0 0] and the recovery pixel becomes white. Since the probability of restoring the secret pixel from a single share is 50%, the attacker cannot reveal any information about a secret image. Because the (2, 2)-EVCS encodes a secret pixel with subpixels, the size of generated shares is four times that of the original image. In the next section, we will propose an expansion-free EVCS mechanism.

As shown in Algorithm 1, we first propose a block-wise halftone method (called gray_level) to divide a gray-level image into *n* nonoverlapping black and white pixel blocks *B*_*i*_, *B*_*i*_∩*B*_*j*_=∅,  for Δ 1 ≤ *i* ≠ *j* ≤ *n*. *B*_*i*_ and halftoned blocks *B*_*h*_ are the same in size. The number of black pixels in *B*_*i*_ and *B*_*h*_ must satisfy the following: the number of black pixels in *Bi*=*s*_*l*_/(*s*_*b*_+1) × (*s*_*l*_ − ∑*Bi*/255)Δ, where *s*_*l*_ denotes the size of candidate black levels, and *s*_*b*_ denotes the block size. To meet the security condition of EVC, the contrast of halftoned black and white blocks (*B*_*h*_) has to be a uniform probability distribution, which results in contrast loss after halftoning.

As shown in Algorithm 2, we limit the gray level of the source secret block; the superimposed gray level will not exceed the gray level of the secret color block. In the encoding process, a gray image is divided into *n* nonoverlapping black and white pixel blocks *B*_*i*_, *B*_*i*_∩*B*_*j*_=∅,  for Δ 1 ≤ *i* ≠ *j* ≤ *n*. *B*_*i*_ and *B*_*h*_ both are of the same size. If there is no restriction on the grayscale during halftoning, if there are three black pixels in the source color block and only two color blocks in the secret color block, the target secret color block cannot be superimposed no matter how it is arranged. Because our block and halftoned blocks are completed independently before encryption, it will not destroy the security of EVCS. Every pixel combination may appear in the basis matrix, so a single participant cannot infer the secret pixel according to the pixel arrangement he holds. The secret image can only be restored when enough participants show their shares. For the (2, 2)-EVCS, if the pixel arrangement held by the other party is complementary to its own, all black pixels will be superimposed, while if the pixel held by the other party is the same as its own, half black and half white gray pixels will be intelligently superimposed. On the other hand, the proportion of black and white pixels in each submemory is fixed, so the whole submemory will not reveal secret image information.

### 3.2. The Recognition of Biomedical Images Recovered from EVC

At present, deep learning methods have achieved great success in the medical field. Its recognition accuracy has exceeded human. The scheme based on VC proposed in this paper should also have high recognition accuracy. However, the sample data recovered from VC is mixed with noise signals, which may affect the accuracy of feature recognition. Therefore, how to propose a new embedding method for VC image restoration and maintain a high accuracy will be another key problem to be solved.

When it is impossible to study an object directly, we can collect a large number of behavior samples of the object and then use a large-scale neural network to approximate the characteristics of black-box objects. Based on the principle, the deep learning method represented by CNN has achieved great success in the field of computer vision through massive data and powerful computing resources. The deep learning method does not need to build a series of complex equations. It can automatically learn the implicit relationship between input features and output targets directly based on historical data and use this relationship to predict unknown data. In a high-precision neural network model for images, data is converted into corresponding weights in the network.

Given the recent success of deep learning methods, we hope to use these methods to solve the problem of image signal interference caused by the introduction of VC. Most neural network models are aimed at specific tasks. Although the best results can be obtained in specific data sets, the performance of the model tends to decline when it is applied to new tasks. Therefore, it takes a lot of computing power to train the network repeatedly for different data sets.

Using the transfer learning method, these weights can be extracted and transferred to other neural networks (such as the restored image mixed with noise signals). Through transfer learning, the learned model parameters can be shared with the new model in a specific way, to speed up and optimize the learning efficiency of the model and avoid learning from zero. Therefore, we first use the pretrained neural network model to generalize and train a softmax classifier on the training data and then fine-tune the weights of the last layer or layers on the data set of a single sample learning task. To avoid affecting the weight information learned by the model, we can freeze the pretrained models (such as ResNet) on data sets such as ImageNet, add several full connection layers at the end of the network, and embed the images restored by VC as training sets, to obtain a high-precision neural network model efficiently. When used as a classification task, the model selects the image class ID most similar to the embedding image in the training set as the output [27].

The framework of a high-precision medical image recognition network based on VC is shown in Figure 3. The input of the network to be trained is three pairs of restored images. The same neural network is used to extract the features of three images to obtain three embedding vectors and then input them into the triple function to calculate the loss. Finally, the backpropagation algorithm is used to update the model parameters according to loss, until a stable neural network model is obtained. After training, we convert the generated template data into binary two-dimensional vectors and then use VCs to store the template in multiple databases. Different from the feature image, the template data does not need to consider the vulnerable problem in the transmission process and can be directly stored by noise image sharing. During image recognition, we firstly generate triplet image pairs and then output the embedding distance between positive, negative, and anchor images. After converting the distance into a probability model, the results of feature recognition and verification can be obtained.

In the process of user registration, the biomedical recognition system uses the EVCS method proposed in this paper to split the private biomedical data into two or more substores and discard the original data. Then shares are stored in two or more different database servers. The private data will not be disclosed to anyone's server unless multiple servers collude. By processing the existing samples one by one, a training dataset for VC can be generated.

In the training process, we directly transfer the corresponding structure and weight to the training of the medical restoration image recognition network by using the model pretrained on large datasets. By removing the original output layer, the pretraining model can be used as a feature classifier. We regard the rest of the whole network as a softmax classifier and apply it to the training of the damaged face image restored by block halftoning technology. We embed the sample and its positive and negative triplets into a low-dimensional vector and then calculate the training loss by using triplet loss until a stable neural network model is obtained.

In the process of authentication, the feature recognition system initiates the transmission request of corresponding shares to database servers. Once the classification recognition or similarity matching is completed, the reconstructed secret image is discarded. In the whole process of registration and identification, the original secret image will be reconstructed only after being authenticated when it is used, and other moments will be stored in separate databases in the form of shared storage. Because of the use of VC, it is theoretically impossible to extract private biomedical information from a single database, so the whole process will not reveal biomedical information.

## 4. Experiments and Results

In this section, we will make a detailed evaluation of the quality of restored images, the encryption efficiency, and the recognition accuracy of decrypted datasets of the proposed new data model. Based on the TensorFlow framework [28], we developed a prototype system of privacy protection for medical images for testing using Python language.

With the proposed limited gray-level halftone method, we can generally transform any existing (*k*, *n*)-EVCS for gray-level images into an expansion-free scheme without affecting the contrast. As shown in Figure 4(b), all five gray levels may appear in the halftone image generated by error diffusion technology, so the generated halftone image is most similar to the original image in Figure 4(a). However, to ensure that the gray levels of the source secret blocks after halftoning are superimposed to meet the gray-level requirements of the secret blocks, we only use limited gray levels in the block halftoning set and fix the proportion of black and white pixels in each color block.  Figure 4(c) uses 4 gray levels (1, 2, 3, 4), while Figure 4(d) only uses two gray levels (3, 4). This means that if Figure 4(d) is divided into nonoverlapping (2, 2) color blocks, the number of black pixels can only be 3 or 4. Because the color block arrangement with 4, 3, and 2 white pixels is deleted, the quality of the restored image is degraded, and it can be seen that the restored image is darker. But we can still see the features of medical images in Figures 4(c) and 4(d). After the block halftoning of the secret image and the cover image is completed, we can rearrange the pixels of the halftone source color block according to the secret color block by combining the existing EVCSs [29].

As shown in Figure 5, (a) is the original secret image, and (c) and (f) are original cover images. We use the two cover images to transmit the secret image, secretly and publicly. Before encryption, we first preprocess these three images with the proposed gray_level method to obtain limited-halftoned images (b), (d), and (g). Then we can encrypt the image (b) block-by-block based on the existing EVCSs to generate two encrypted cover images (e) and (h). Although there is contrast loss, the original cover images are still visible in the two images. The decrypted image (i) is obtained by simply overlaying the two images, that is, performing a Boolean AND operation. The proposed scheme keeps the printable characteristic of VCS.

We then test the performance of the proposed architecture on the classical BreakHis (Breast Cancer Histopathological Dataset) [30]. Breast cancer is one of the most common cancers among women in the United States, with more than 2 million new cases each year, according to the World Cancer Research Fund. Breast cancer detection is a very time-consuming task due to the reliance on the expertise of pathologists. With rapid advances in machine learning and deep learning, computer-aided diagnosis can provide useful support for pathologists. The BreakHis consists of 7,909 microscopic images of breast tumor tissue collected in 82 patients using various magnification factors including 40x, 100x, 200x, and 400x. BreakHis contains 2,480 benign and 5,429 malignant samples (700 × 460 pixels, 3-channel RGB, 8-bit depth in each channel, PNG format). We use class 0 to indicate malignant samples and 1 to indicate benign samples in all experiments.

Figure 6 shows the performance comparison between our novel VC scheme and Lee and Chiu [22] scheme. Although both schemes can realize user-friendly encryption without pixel extension, Lee's scheme uses optimization schemes including simulated annealing, which leads to low efficiency of encryption sharing generation. With our scheme, we can directly select the basic matrix blocks from the candidate matrices and place them in the corresponding positions of shares to complete the encryption. So, our encryption efficiency is about 10 times faster than Lee's.

We select images with 40x magnification as training and test sets for simplicity in the experiment, where 70% are used as training sets and 30% as test sets. As shown in Table 1, the accuracy of our methods is over 95%, while the accuracy in the originally published paper is only 83.8%. Despite the loss in our images, the accuracy is much better than Fabio's method [31], which is due to the new model ResNet [32] we used. The experiment shows that the powerful generalization of transfer learning allows prediction performance on lossy datasets to exceed that of the original dataset.

Figures 7 and 8 show the ROC (Receiver Operating Characteristic) curves of the BreakHis dataset from normal and recovery images with various magnification factors. The macroaverage metric will calculate the metric of each class independently and then take its average, so all classes will be treated equally, whereas the microaverage will summarize the contributions of all classes and calculate the average metric. It can be seen that AUCs (Area Under Curve) are all above 0.99 for different magnification of datasets.

To eliminate the effect of sample distribution on experimental results, we compute the sensitivity (recall) and precision measures, where sensitivity indicates the effectiveness of detecting cancer in a population with cancer and precision indicates the extent to which the test is positive in a population without the disease. For the ideal computer-aided diagnostic method, we want as few patients as possible to go undetected (high sensitivity) and as few nonpatients as possible to undergo further diagnostic testing (high specificity). The *f*1-score is the harmonic mean of the sensitivity and specificity.

Table 2 shows a performance comparison between the normal dataset and the dataset recovered from the proposed EVC. The prediction accuracy reaches 0.99 for the 100x magnification factor. However, it is worth noting that the accuracy does not increase with the increase of factors but even decreases. This is because, in the case of consistent image size, too small scale disperses the learning of features, while too large scale may lose some features. This experiment shows that, for medical images, the sampling factor is crucial to recognition accuracy. The metrics in the recovered dataset are lower than those of the original images, while the performance degradation is not significant, all within 5%. This is because although medical images consist of more complex patterns than normal images, this encryption is equivalent to adding global white noise to the image. It is a lossy transformation and will not destroy the characteristics of medical images. A small amount of global noise will not affect the automatic learning and extraction of features in the image using CNN.

We further evaluate the proposed algorithm on the LFW (Labeled Faces in the Wild) dataset to verify the universality of the proposed method. The LFW face dataset is the de-facto benchmark for face verification. Biomedical authentication is a technology that uses human biomedical characteristics (such as a face) for identity authentication. It is strongly bound to the user's identity in the network environment, which makes up for the defects of the traditional authentication method based on cryptography. Due to the uniqueness and persistence of biomedical characteristics, once leaked, it will cause permanent losses. The development of artificial intelligence technology has promoted the wide use of biomedical authentication technology, but it has also aggravated the concern of society about privacy leakage of biomedical features.

Our method also can preserve the privacy of biometrics like LFW when transmitting on a public network. As shown in Table 3, the proposed model can archive results of more than 0.93. Especially for the accuracy, it reaches 0.97. The reason why our model can surpass the medical dataset in the face dataset is that the face data set has a larger sample size (more than 13000). Second, compared with medical images, face images have more features (such as eye, mouth, eyebrows, etc.) that can be extracted.

### 4.1. Security Analysis

The proposed schemes ensure the confidentiality of images by a secret-sharing algorithm when constructing shares. Therefore, it is impossible to access the secret from shared images. A single share or less than the threshold will not reveal any secret information. As shown in Figure 5, shares look like natural images and will not reveal secrets individually. We perform the preprocessing operation before encrypting. The preprocessing process, which does not involve the secret image, is only related to the current image. So, the process of preprocessing will not disclose any part of a secret image. In the next encryption process, we base on the existing EVCS mechanism [29], so the encryption process is also secure. With the proposed limited gray-level halftone method, we can generally transform any existing (*k*, *n*)-EVCS for gray-level images into an expansion-free scheme. The difference is that we adopt the mechanism of block encryption to encrypt the image, while in the original EVCS, the image is encrypted pixel-by-pixel. We interpret blocks containing 2 or 3 black pixels as white pixels and blocks containing 3 or 4 black pixels as black pixels so that the encryption process can reuse the original basis matrices. Since the contrast of the reinterpreted black and white color blocks still satisfies condition (iii) in Section 3, we can still see the information from encrypted cover images as well as the recovery image according to the halftone effect of images.

## 5. Conclusion

Sophisticated communications schemes are required for medical data to communicate effective implementation capabilities. In this paper, we proposed an efficient and key-free data protection model based on VC for medical data transmission and template storage. To protect the privacy of sensitive biological features, we decompose the secret image into two meaningful images to safely store the feature template data. Each shared image does not display any information about the original image, and the secret image can only be displayed when two images are available at the same time. Triplet loss is used as the loss function of feature recognition, which is combined with transfer learning to enhance the recognition performance of noise image recovery from EVCS. The experimental results and comparative analysis show that our method preserves the recognition performance and accuracy while protecting the data.

In the future work, we will combine the characteristics of OR and XOR operations to propose a novel VCS that can perfectly restore the image with low computing power dependence and eliminate the image expansion without computing power dependence, to expand the application scope of VC. Aiming at the noise interference of the restored image by VC, we will use the progress of the deep neural network in image denoising and propose a denoising neural network for VC to improve the quality of the restored image.

## Figures and Tables

**Figure 1:** Illustration of the encryption and decryption of a 2X2-VCS.

**Figure 2:** The encryption and decryption flow for a (2, 2)-EVCS.

**Figure 3:** High-precision medical image recognition network based on VC.

**Figure 4:** The halftoned images with error diffusion and our gray_level methods. (a) Original image. (b) The halftone image with all gray levels. (c) The halftone image with 4 gray levels. (d) The halftone image with 2 gray levels.

**Figure 5:** The experimental result for the proposed EF-EVCS: (a), (c), and (f) are the original secret (lena), cover 1 (peppers), and cover 2 (butterfly) images; (b), (d), and (g) are corresponding limited-halftoned images; (e) and (h) are encrypted images for sharing; (i) is the recovery image by stacking (e) and (h).

**Figure 6:** Comparison of encryption performance of two EVCS (our and Lee's).

**Figure 7:** The ROC curves and AUCs of the BreakHis dataset from normal images with magnification factors including 40x (a), 100x (b), 200x (c), and 400x (d). We use class 0 to indicate malignant samples and 1 to indicate benign samples.

**Figure 8:** The ROC curves and AUCs of the BreakHis dataset from recovery images with magnification factors including 40x (a), 100x (b), 200x (c), and 400x (d). We use class 0 to indicate malignant samples and 1 to indicate benign samples.

**Algorithm 1:** Limited gray-level halftoning algorithm (gray_level).

**Algorithm 2:** An expand-free EVCS algorithm.

**Table 1:** Comparison of recognition performance among datasets from our proposed EVCS, Fabio's method, and normal datasets.

Metric	EVCS	Fabio's method	Normal
Accuracy	0.94	83.8	0.97
Recall	0.93	—	0.96
Precision	0.96	—	0.98
*f*1-score	0.93	—	0.97

**Table 2:** Performance comparison between the normal dataset and dataset recovered from VCS.

Type	Precision		Recall		*F*1-score		Accuracy		Support
	EVC	Normal	EVC	Normal	EVC	Normal	EVC	Normal	
Malignant (0, 40x)	0.94	0.97	0.99	0.99	0.97	0.98	0.95	0.97	2349
Benign (1, 40x)	0.98	0.98	0.87	0.95	0.93	0.97			1160
0, 100x	1.00	1.00	0.99	0.99	0.99	0.99	0.99	0.99	2386
1, 100x	0.98	0.98	0.99	0.99	0.99	0.99			1182
0, 200x	1.00	0.99	0.98	0.99	0.99	0.98	0.98	0.99	2335
1, 200x	0.95	0.96	1.00	0.98	0.98	0.99			1114
0, 400x	1.00	1.00	0.97	0.95	0.99	0.97	0.96	0.97	2080
1, 400x	0.95	0.91	100	1.00	0.97	0.95			1059

**Table 3:** Recognition performance on the face dataset (LFW).

Metrics	Accuracy	Precision	Recall	*F*1-score
LFW	0.97	0.96	0.93	0.93

## Data Availability

The data used to support the findings of this study are available from the corresponding author upon request.
